# Structural and Functional Annotation and Molecular Docking Analysis of a Hypothetical Protein from *Neisseria gonorrhoeae*: An In-Silico Approach

**DOI:** 10.1155/2022/4302625

**Published:** 2022-09-05

**Authors:** Lincon Mazumder, Md. Rakibul Hasan, Kanij Fatema, Md. Zahirul Islam, Sanjida Khanam Tamanna

**Affiliations:** Department of Microbiology, Jagannath University, Dhaka 1100, Bangladesh

## Abstract

**Background:**

Worldwide, *Neisseria gonorrhoeae*-related sexually transmitted infections (STIs) continue to be of significant public health concern. This obligate-human pathogen has developed a number of defenses against both innate and adaptive immune responses during infection, some of which are mediated by the pathogen's proteins. Hence, the uncharacterized proteins of *N. gonorrhoeae* can be annotated to get insight into the unique functions of this organism related to its pathogenicity and to find a more efficient therapeutic target.

**Methods:**

In this study, a hypothetical protein (HP) of *N. gonorrhoeae* was chosen for analysis and an in-silico approach was used to explore various properties such as physicochemical characteristics, subcellular localization, secondary structure, 3D structures, and functional annotation of that HP. Finally, a molecular docking analysis was performed to design an epitope-based vaccine against that HP.

**Results:**

This study has identified the potential role of the chosen HP of *N. gonorrhoeae* in plasmid transfer, cell cycle control, cell division, and chromosome partitioning. Acidic nature, thermal stability, cytoplasmic localization of the protein, and some of its other physicochemical properties have also been identified through this study. Molecular docking analysis has demonstrated that one of the T cell epitopes of the protein has a significant binding affinity with the human leukocyte antigen HLA-B∗15 : 01.

**Conclusions:**

The in-silico characterization of this protein will help us understand molecular mechanism of action of *N. gonorrhoeae* and get an insight into novel therapeutic identification processes. This research will, therefore, enhance our knowledge to find new medications to tackle this potential threat to humankind.

## 1. Introduction

*N. gonorrhoeae*, the etiological agent of Gonorrhea, first isolated in 1878, belonging to the *Neisseriaceae* family [1, 2], is a gram-negative, 0.6-1 micrometer in diameter [3], encapsulated bacterium [4]. It is fastidious [5], non-acid fast [6], oxidase-positive [7], and non-spore-forming in nature [8]. In addition, it is a non-motile [9] and obligate-human pathogen [10] that can thrive aerobically or anaerobically in the presence of nitrite [11]. These diplococci, kidney-shaped bacteria infecting both men and women can cause the sexually transmitted disease (STD) named gonorrhea [12, 13]. Every year, 87 million new infections are being reported for this quick-spreading contagious disease. This STD has already emerged as a major problem in low- and middle-income countries in Africa, Asia, Latin America, and the Caribbean [1, 5, 12]. Gonorrhea can be asymptotic or develop with symptoms. It can manifest as urethritis in men, with symptoms such as epididymitis, urethral stricture, and prostatitis. In women, it might manifest as urethritis or cervicitis, with symptoms including tubal infertility, chronic pelvic discomfort, severe pelvic inflammatory disease sequelae, and ectopic pregnancy [3, 14]. Oropharyngeal and anorectal gonococcal infections can be transmitted from one person to another through kissing and during oral-anal intercourse. Furthermore, gonorrhea can be caused by contamination via cervical fluids [14, 15]. However, there is still no effective treatment for gonococci and even no gonococcal vaccination is available yet. To make the situation worse, *N. gonorrhoeae* has been found resistant to several antimicrobial drugs such as penicillins, tetracyclines, sulphonamides, fluoroquinolones, macrolides, azithromycin, and ceftriaxone [12, 16, 17]. Hence, WHO recommends azithromycin and ceftriaxone as a dual therapy for the time being against this disease [12]. All these things have now made the discovery of novel antibacterial drugs and the development of alternative therapies a crying need for combating this disease [18].

The genome size of *N. gonorrhoeae* varies from strain to strain, about 2001+/-197 kbp [19]. For example, the genome of *N. gonorrhoeae* NCCP11945 contains 2232.025 kbp in one circular chromosome that encodes 2662 predicted open reading frames and 4153 bp that codes 12 predicted ORFs [20]. Additionally, *N. gonorrhoeae* is known to encode several proteins with unknown functions, known as hypothetical proteins (HPs). HPs are considered to be expressed in an organism, but there is no experimental and chemical proof of their existence [21–23]. In most genomes, HPs cover approximately half of the protein-coding regions, but these proteins' roles are yet to be discovered [21, 24, 25]. Although there is no empirical evidence for the existence of these proteins, they can be predicted to be generated from an open reading frame (ORF) [23, 24]. As a result, the annotation of the functions of hypothetical proteins has become increasingly popular [25]. The hypothetical proteins can be categorized as uncharacterized protein families (UPF) as well as the domain of unknown functions (DUF) [23]. Uncharacterized protein families (UPF) have been experimentally confirmed to exist, although they have yet to be identified or connected to a known gene. On the other hand, DUFs are proteins that have been found experimentally but have no known functional or structural domains [23]. Even though they have not been characterized, elucidating their structural and functional secrets can lead to the identification of new domains and motifs, pathways and cascades, structural conformations, protein networks, etc. [21, 22]. These are crucial in understanding biochemical and physiological pathways, for example, in identifying pharmaceutical targets [21, 22, 25] and providing early detection and advantages for proteomic and genomic studies [21]. It is now easier to analyze hypothetical proteins utilizing a variety of bioinformatics tools that provide benefits such as 3D structural conformation prediction, identification of new domains and pathways, phylogenetic profiling, and functional annotation [22, 23].

The purpose of this study is to characterize a hypothetical protein F0T10_13280 (plasmid) of *N. gonorrhoeae* with an integrated computational approach, with previously validated tools and databases, to get an insight into the HP's physical and structural information along with its potential functions. Potential role of this HP in plasmid transfer, cell cycle control, cell division, and chromosome partitioning may give insight into the pathogenic flexibility of *N. gonorrhoeae*. Analyzing the phylogenetic relationship between this HP and other proteins, physicochemical properties analysis, prediction of the HP's location in the cell, analysis of the secondary and tertiary structure, prediction of the potential function of the HP, and evaluation of the active sites are some of the main focuses of this research. Finally, this research also aims to design an epitope-based peptide vaccine and validate it with a molecular docking study.  Figure 1 illustrates the complete workflow and tools used in this study.  Table 1 depicts the entire framework, which includes all the tools used to annotate the structural and functional properties of HP of *N. gonorrhoeae.* A preprint of this research has previously been published by Mazumder et al. [26]

## 2. Materials and Methods

### 2.1. Sequence Retrieval and Phylogeny Analysis

The amino acid sequence (accession No. QIH20856.1) was selected by searching the NCBI protein database for HP of *N. gonorrhoeae.* The sequence was obtained in FASTA format. To identify sequence similarity, BlastP [27] was performed. MUSCLE v3.6 [28] was used to perform multiple sequence alignment. Phylogenetic analysis was carried out using MEGA X [29].

### 2.2. Physicochemical Properties Analysis

The physicochemical properties of the target protein sequence were investigated using ExPASy's ProtParam program [30]. The molecular weight, atomic composition, estimated half-life, theoretical isoelectric point (pl), extinction coefficient, amino acid composition, aliphatic index, stability index, the total number of positive and negative residues, and grand average of hydropathicity (GRAVY) were all analyzed using this tool.

### 2.3. Subcellular Localization Prediction

It is crucial to know the subcellular localization of proteins in order to comprehend their functions [31] entirely. Computer analysis helps in the discovery and localization of adhesion-like intercellular proteins [32]. In the last few decades, several computational tools have been developed that can efficiently determine and synthesize ORFs of various proteins (mitochondrial, cytoplasmic, nuclear, or extracellular) to convert them into potential vaccine candidates. However, vaccine candidates should be free of membrane or cytoplasmic localization [33]. CELLO v.2.5 [34] was first used to recognize the subcellular localization of hypothetical protein F0T10_13280 (plasmid) of *N. gonorrhoeae*. PSORTb v3.0.3 [35] was further used to anticipate subcellular location. To cross-check the results, we used PSLpred [36], a web server for predicting the subcellular localization of gram-negative bacterial proteins.

### 2.4. Secondary Structure Prediction

Secondary structure predictions of the hypothetical protein were performed using the SOPMA server [37]. The PSIPRED server [38] was also used to ensure the accuracy of the SOPMA results.

### 2.5. 3D Structure Prediction and Quality Assessment

HHpred server [39] provided a 3D model of the protein. The YASARA server [40] (http://www.yasara.org/minimizationserver.htm) was used to accomplish energy minimization. To visualize the final model and perform structural analysis, PyMOL v2 [41] was employed. The SAVES server's (https://services.mbi.ucla.edu) quality assessment tools were used to assess the predictability of the hypothetical protein's projected 3D structural model. The Ramachandran plot was built using the PROCHECK [42] tool to visualize the backbone dihedral angles of amino acid residues. With the help of the ERRAT server [43], the quality of the protein 3D structure was evaluated. The Verify 3D server [44] was used to check whether an atomic model (3D) was compatible with its amino acid sequence and compare the results to standard structures.

### 2.6. Functional Annotation

In order to make exact and reliable functional predictions of the HP, we used a variety of tools. INTERPRO [45], MOTIF [46], Pfam [47], and the conserved domain database of NCBI [48] are the databases and tools being used for this requirement.

### 2.7. Active Site Detection

For active site assessment and structure-based ligand design, the shape and size of protein pockets and cavities are crucial. The computed atlas of surface topography of proteins (CASTp) was utilized in this experiment to detect possible binding sites, pockets, and cavities from the 3D structure of the target protein [49].

### 2.8. Prediction of CTL Epitope and MHC I Binding Allele Analysis

In order to design an epitope-based vaccine against the hypothetical protein, cytotoxic T lymphocytes (CTL) prediction was performed using the NetCTL server [50]. The threshold parameter was set to 0.4 with 0.89 sensitivity and 0.94 specificity. To analyze the MHC I binding alleles, all CTL was evaluated with the immune epitope database (IEDB) utilizing the SMM method [51]. The MHC I alleles for which the epitopes showed higher affinity (IC50< 500 nM) were selected for further analysis.

### 2.9. Epitope Selection for Docking and Epitope Prioritization

Among all the CTL epitopes, one epitope was selected based on its interaction with the maximum number of MHC I binding alleles. The suitability of this epitope for vaccine construction was cross-checked with VaxiJen 2.0 [52], Toxinpred [53], and AllerTOP 2.0 [54] servers to investigate the antigenic, allergenic, and toxicity properties, respectively. The threshold parameter of the VaxiJen 2.0 server was set to 0.4, and all the parameters of the Toxinpred and AllerTop 2.0 server were set to default.

### 2.10. Peptide Designing and Docking Analysis

The three-dimensional structure of the epitope was constructed with the APPTEST server [55]. APPTEST server is a peptide tertiary structure prediction tool that predicts peptide structure using a neural network architecture and simulated annealing methods. A molecular docking experiment was performed to scrutinize the binding interaction between the epitope and receptor molecule. The crystal structure of HLA-B∗15 : 01 (PDB ID – 1xr8) was retrieved from the RCSB database [56] to perform docking analysis. The docking analysis between the peptide (ligand) and human receptor HLA-B∗15 : 01 was performed using the AutoDockVina tool [57]. The grid box size of the AutoDockVina tool was kept at 12.702, 31.843, and 18.307, respectively, for *X*, *Y*, and *Z*. The binding interactions and residues in the interacting surface between the peptide and receptor were investigated with Discovery Studio 2021 [58].

## 3. Results and Discussion

### 3.1. Sequence and Similarity Information

We selected a hypothetical protein (accession no. QIH20856.1) from the organism *N. gonorrhoeae*. This hypothetical protein contains 478 amino acids. The amino acid sequence for this protein was selected from the NCBI database and obtained in FASTA format. BlastP was performed to verify sequence similarity. The non-redundant protein sequences (nr) database (Table 2) and the UniProt/Swiss-Prot (SwissProt) database (Table 3) were examined to identify sequence similarity with other known proteins by utilizing BlastP. The HP exhibits similarities with other MobA/MobL family proteins, according to the non-redundant protein sequence database. A phylogenetic tree showing the phylogenetic relatedness among the sequences obtained from the non-redundant database was constructed using the MEGA X program by neighbor-joining method with a bootstrap replication of 1000, shown in Figure 2.

### 3.2. Physicochemical Properties

According to the ExPASy ProtParam server, the protein's physical properties (Table 4) revealed that it includes 478 amino acids. The most prevalent amino acids in the composition were Ala (37), Arg (30), Asn (23), Asp (26), Cys (3), Gln (47), Glu (55), Gly (20), His (10), Ile (26), Leu (34), Lys (53), Met (7), Phe (17), Pro (11), Ser (28), Thr (15), Tyr (20), Trp (5), and Val (11). Its molecular weight is 56206.84 Dalton. The hypothetical protein has an instability index of 45.45, indicating that it is a stable protein. The numbers of negatively charged (Asp + Glu) and positively charged (Arg + Lys) residues were calculated to be 81 and 83, respectively. The aliphatic index was found to be 63.37, indicating that the protein is stable across an extensive temperature range. The protein's GRAVY score of 1.179 suggested that it is water-soluble (hydrophilic). The protein's pI was calculated to be 8.07, indicating that it is acidic (pH 7) in nature. The molecular formula of the HP was C2461H3884N716O774S10. In mammalian reticulocytes (in vitro), yeast (in vivo), and *E. coli*, the putative protein's half-life was calculated to be 30 hours in mammalian reticulocytes (in vitro), > 20 hours in yeast (in vivo), and> 10 hours in *E. coli* (in vivo).

### 3.3. Subcellular Localization Prediction

The environments in which proteins operate are determined by their subcellular localization. Protein subcellular localization is crucial for understanding protein function. Predicting an unknown protein's subcellular localization also provides valuable information about genomic annotation and drug design [31]. The prediction of an unknown protein's subcellular localization can be used to understand disease mechanisms as well as to develop drug or vaccine targets in a given pathogen genome [59]. The cytoplasmic proteins may serve as less suitable potential therapeutic targets, whereas surface membrane proteins are thought to be effective vaccine targets [33, 60]. In our study, we have found our protein as cytoplasmic according to the result of the CELLO. The localization score from CELLO was found to be 1.680. PSORTb v3.0.3 and PSLpred were used to verify the result. PSORTb v3.0.3 also identified the protein to be cytoplasmic, and the score was found to be 8.96. According to the PSLpred, the protein was also predicted as a cytoplasm-resident protein with a score of 64.47.

### 3.4. Secondary Structure Prediction

The secondary structure (helix, sheet, turn, and coil) aids in providing information on each amino acid's conformation. Protein secondary structure prediction can be used to predict tertiary structure and the primary sequence and tertiary structure are linked by it [61]. Though protein secondary structure prediction is an essential first step toward predicting tertiary structure, it also provides details on protein activity, interactions, and functions. Alpha helices were found to be the most frequently occurring structure in the HP while examined by SOPMA (69.87 percent) (Figure 3). The random coil was seen at 19.67 percent, followed by the extended strand at 5.65 percent. In addition, beta-turn was found to be 4.81 percent. We cross-checked the results using PSIPRED, and a similar result was revealed (Figure 4).

### 3.5. Homology Modelling, Quality Assessment of the 3D Model, and Visualization

The 3D structure of the protein is highly related to its function. It also helps to predict the binding sites and active sites of the protein, which may contribute to design an effective vaccine against that pathogen. The 3D structure of the HP was obtained from HHpred server using homology modelling. By lowering the energy from -48,361.0 kJ/mol to -11487.9 kJ/mol, the YASARA energy minimization server made the model structure more stable. The 3D structure of the protein was developed by PyMOL v2 (Figure 5). A variety of quality assessment tools were employed to determine how reliable the protein's predicted 3D structural model was. PROCHECK's Ramachandran plot analysis, Verify3D, and ERRAT verified the protein's 3D structure. According to the Ramachandran Plot Statistics (Figure 6(a)), the model was thought to be acceptable, with 93.6 percent residues in the most favored regions (Table 5), and it was 90.8 percent before energy minimization. Utilizing the ERRAT and Verify3D programs, the initial structural model was assessed for 3D structure errors. After energy minimization, ERRAT determined that the model was of good quality with an overall quality factor of 95.556 (Figure 6(b)), whereas it was 78.453% prior to energy minimization. After energy minimization, The Verify3D showed that (Figure 6(c)) 96.30 percent of the residues have averaged 3D-1D score >= 0.2, indicating that the model's environmental profile is good. A comparison of all the quality factors of the predicted structure before and after energy minimization is summarized in Table 6.

### 3.6. Functional Annotation

Using the NCBI's conserved domain search tool, two functional domains of the HP were identified. The domain detected in the HP belongs to the MobA/MobL protein family (accession No. pfam03389). This family includes the MobA protein from the *E. coli* plasmid RSF1010 and the MobL protein from the *Thiobacillus ferrooxidans* plasmid PTF1. These are mobilization proteins, which are required for particular plasmid transfer. Smc or chromosomal segregation ATPase is another superfamily that involves cell cycle control, cell division, and chromosome partitioning. Plasmid transfer, cell division, cell cycle regulation, and chromosomal partitioning are essential aspects of genetic engineering and the biotechnological approach. Cell cycle regulation is critical for cell survival and proliferation. Lack of cell cycle maintenance can result in harmful mutations, leading to cell death and cancer [62]. This result was also cross-checked using INTERPRO, MOTIF, and Pfam. All produced similar findings, with positions ranging from 23 to 211 amino acid residues and an *e*-value of 3.5e-29.

### 3.7. Active Site Detection

Several studies have documented that the discovery and identification of active sites on proteins are becoming highly significant. The position of the active site on a protein is pivotal for a variety of purposes, including structural identification, functional site comparison, molecular docking, and de novo drug creation [26]. Since the computed atlas of surface topography of proteins (CASTp) just employs the C*α* atoms to represent the protein structure, it is quick and appropriate for usage with models and unreliable structures. The geometric potential is a concept to quantitatively describe the shape of the protein structure, which can be affected by the overall form of the structure and individual residue's surroundings. About 85% of known binding sites may be reliably predicted by CASTp with above 50% residue coverage and 80% specificity, and it often uses the geometric potential for this purpose [63]. Hence, the CASTp server was used in this study to examine the protein's active site. The region involved in active site formation is illustrated in Figure 7. The CASTp server revealed that the active site of the protein had 16 amino acid residues, with the best active site located in regions with 63.924 and a volume of 57.845.

### 3.8. Prediction of CTL Epitope and Analysis of the MHC I Binding Alleles

The majority of vaccinations now in use are based on B cell immunity. However, any foreign particle can eventually avoid the antibody memory response due to antigenic drift. Therefore, T cell epitope-based vaccines have been promoted since the T cell immune response frequently results in long-lasting protection. A powerful immunological response against the infected cell can be produced by the host via CD8+ T cells [64]. Hence, T cell epitope prediction was performed with the most used computational server, NetCTL 1.2. The NetCTL server anticipated the 13 effective T cell epitopes from the selected protein sequence, such as QSAQAKNDY, LTDKNQGFL, GMEVEITQY, DSGSNKLPY, HTDKNNHNP, QANQALEQY, KQAQGMGKY, FAEDNPQEF, NQALEQYGY, LDDLQFSGY, AIYHLNVRY, DLQRIQGDY, and TVDSGSNKL with a specificity score of 0.940 and a sensitivity score of 0.89. The MHC I alleles for which the epitopes showed higher affinity (IC50 <500 nM) are shown in Table 7.

### 3.9. Epitope Selection for Docking and Epitope Prioritization

Among the 13 T cell epitopes, the epitope AIYHLNVRY was found to interact with the highest number of MHC I alleles and was selected for vaccine design. This epitope interacted with 5 MHC I binding alleles, including- HLA-A∗30 : 02, HLA-A∗32 : 01, HLA-B∗15 : 01, HLA-A∗03 : 01, and HLA-A∗11 : 01. A vaccine candidate epitope must meet a number of requirements and our projected epitope met every requirement. The initial criterion requires that the epitope must induce an immunogenic response in the host. The VaxiJen 2.0 antigenic analysis tool was used to determine if the epitope had caused an immunogenic response in the host. Upon the analysis with this tool, it has been identified that the epitope is a putative antigen (antigenicity score 1.5783). Testing for toxicity is another crucial step in the creation of a vaccine. ToxinPred server identified the epitope as a non-toxic epitope. However, one of the main challenges to the creation of vaccines is allergenicity. Most vaccinations trigger an allergic immune response by inducing type 2 T helper (Th2) cells and immunoglobulin E [65]. AllerTOP 2.0 server identified the epitope as a non-allergen protein. All these results have identified the epitope as a suitable vaccine candidate.

### 3.10. Molecular Docking Analysis

To evaluate the proposed epitope vaccine's affinity for the human leukocyte antigen HLA-B∗15 : 01, ligand-receptor docking has been performed. The docking analysis with AutoDockVina tool has revealed that the predicted epitope produced a total of nine hydrogen bonds with the residue Tyr9, Arg8, Val7, Ala1, Tyr3, Ile2, Asn6, Leu5, and His 2. The binding energy between the epitope and HLA-B∗15 : 01 receptor was found to be -7.5 kcal/mol. Strong hydrogen bonds and the docked complex's lowest energy value demonstrate a stable connection between the ligand and the receptor molecule. The three-dimensional structure of the peptide and the binding interactions of the peptide and HLA-B∗15 : 01 after docking analysis are visualized and captured with Discovery Studio 2021 and shown in Figure 8.

## 4. Conclusion

Throughout this study, we investigated a hypothetical protein from the bacteria *Neisseria gonorrhoeae* by utilizing several bioinformatics tools. According to our experiment, several physicochemical and functional properties of the studied hypothetical protein have been revealed. Although the cytoplasmic position of this protein makes it less suitable for prospective vaccine design, the molecular docking analysis performed in this study may serve as a foundation for future in-silico vaccine design research, and subsequently, this study will assist other researchers. This study may enhance our understanding of studying the structural and functional research of proteins with unknown functions. Additionally, this research study may subsequently benefit other researchers to do in-silico studies independently. However, as our analysis is based on computational tools and databases, further in vitro and in vivo research is suggested for experimental validation.

## Figures and Tables

**Figure 1:** Complete flowchart of the hypothetical proteins (HPs) annotation process used in this study.

**Figure 2:** Phylogenetic relationship among the hypothetical protein and other similar proteins obtained from the non-redundant database by BlastP search. The evolutionary distances were computed using the Poisson correction method and are in the units of the number of amino acid substitutions per site.

**Figure 3:** Secondary structure model predicted by the SOPMA server.

**Figure 4:** Secondary structure model by PSIPRED server.

**Figure 5:** Predicted 3D structure of the hypothetical protein visualized by PyMOL (before and after energy minimization).

**Figure 6:** (a) The PROCHECK program validated the Ramachandran plot of the predicted structure. (b) Quality factor 95.556 for ERRAT output. Two lines on the error axis represent the level of confidence required to reject areas that exceed the error value. (c) Verify3D prediction outcome showing 96.30% of the residues have averaged 3D-1D score >= 0.2.

**Figure 7:** Active site (red color) of the studied hypothetical protein.

**Figure 8:** Docking analysis revealed by AutodockVina. (a) Three-dimensional structure of the predicted epitope, “AIYHLNVRY” and (b) visualization of binding interactions and residues after the docking of “AIYHLNVRY” with HLA-B∗15 : 01.

**Table 1:** List of bioinformatics tools and databases used in this study for structural and functional analysis of the HP.

S.N.	Tools/server	URL	Function	References
(A) Sequence similarity search				
1	BLAST	http://www.ncbi.nlm.nih.gov/BLAST/	Find similar sequences in protein databases	27
2.	MUSCLE		Multiple sequence alignment prediction	28
3.	MEGA X		Phylogenetic tree analysis	29
(B) Physiochemical characterization				
4.	ExPASy – ProtParam	http://web.expasy.org/protparam/	Used for predicting physicochemical properties	30
(C) Subcellular localization identification				
5.	PSORT B v3.0	http://www.psort.org/psortb/	Predict subcellular localization	35
6.	PSLpred	http://www.imtech.res.in/raghava/pslpred/	Predict subcellular localization	36
7.	CELLO	http://cello.life.nctu.edu.tw/	Predict subcellular localization	34
(D) Secondary structure prediction				
8.	SOPMA	https://npsa-prabi.ibcp.fr/cgi-bin/npsa_automat.pl?page=/NPSA/npsa_sopma.html	Predict the secondary structure of the protein	37
9.	PSIPRED	http://bioinf.cs.ucl.ac.uk/psipred/	Predict secondary structure	38
(E) 3D structure prediction and quality assessment				
10.	HHpred	https://toolkit.tuebingen.mpg.de/tools/hhpred	Detect protein homology	39
11.	YASARA	http://www.yasara.org/minimizationserver.htm	Utilized to increase the stability of the 3D model structure	40
12.	PROCHECK's	https://saves.mbi.ucla.edu/	Used for Ramachandran plot analysis	42
13.	Verify3D	https://saves.mbi.ucla.edu/	Structure verification	44
14.	ERRAT	https://saves.mbi.ucla.edu/	Used to analyze the statistics of nonbonded interactions between different atoms and verify protein structures	43
(F) Functional characterization				
15.	Conserved domain database	http://www.ncbi.nlm.nih.gov/Structure/cdd/wrpsb.cgi	Used to search functional domains in a sequence	48
16.	Pfam	http://pfam.xfam.org/	Family relationship identification	47
17.	INTERPRO	http://www.ebi.ac.uk/interpro/	Used to search InterPro for motif discovery	45
18.	MOTIF	http://www.genome.jp/tools/motif/	Motif discovery	46
(G) Active site identification				
19.	CASTp	http://sts.bioe.uic.edu/castp/	Used to find, outline, and estimate inward surface regions on protein 3D structure	49

**Table 2:** Similar protein obtained from non-redundant protein sequences (nr) database.

Description	Scientific name	Max score	Total score	*E* value	Percent identity	Accession
MobA/MobL family protein [Proteobacteria]	*Proteobacteria*	984	984	0	100	WP_032490546.1
MobA/MobL family protein [Haemophilus parainfluenzae]	*Haemophilus parainfluenza*	978	978	0	99.37	WP_197561055.1
MobA/MobL family protein [Haemophilus haemolyticus]	*Haemophilus haemolyticus*	977	977	0	99.16	WP_140450219.1
MobA/MobL family protein [Neisseria gonorrhoeae]	*Neisseria gonorrhoeae*	936	936	0	96.86	WP_127514845.1
MobA/MobL family protein [Haemophilus parainfluenzae]	*Haemophilus parainfluenzae*	907	907	0	99.11	MBS6191364.1

**Table 3:** Similar protein obtained from UniProt/Swiss-Prot (SwissProt) database.

Description	Scientific name	Max score	Total score	*E* value	Per. Ident	Accession
[*Escherichia coli*]	*Escherichia coli*	219	219	1.00E-62	46.96	P07112.4
[Salmonella enterica subsp. enterica serovar Typhimurium]	Salmonella enterica subsp. enterica serovar Typhimurium	154	154	2.00E-41	41.01	P14492.1
[*Acidithiobacillus ferridurans*]	*Acidithiobacillus ferridurans*	86.7	86.7	3.00E-17	27.91	P20085.1
[*Bifidobacterium longum* NCC2705]	*Bifidobacterium longum* NCC2705	73.2	73.2	2.00E-12	26.32	Q8GN32.1
[*Agrobacterium tumefaciens*]	*Agrobacterium tumefaciens*	65.9	65.9	5.00E-10	24.58	Q44363.1

**Table 4:** ProtParam tool analysis result for the HP of *Neisseria gonorrhoeae* F0T10 13280.

Number of amino acids	478
Molecular weight	56206.84
Theoretical pI	8.07
Total number of negatively charged residues (Asp + Glu)	81
Total number of positively charged residues (Arg + Lys)	83
Formula	C_2461_H_3884_N_716_O_774_S_10_
Instability index (II)	45.45
Aliphatic index	63.37
Grand average of hydropathicity (GRAVY)	-1.179
The estimated half-life is	Thirty hours (mammalian reticulocytes, in vitro). >20 hours (yeast, in vivo). >10 hours (Escherichia coli, in vivo).

**Table 5:** Ramachandran plot statistics of the predicted 3D model for studied protein.

Ramachandran plot analysis	No. (%)
Residues in the most favored regions [A, B, L]	159 (91.9%)
Residues in the additional allowed regions [a, b, l, p]	13 (7.5%)
Residues in the generously allowed regions [-a, -b, -l, -p]	1 (0.6%)
Residues in the disallowed regions	0 (0.0)
No. of non-glycine and non-proline residues	173 (100.0%)
No. of end-residues (excl. Gly and Pro)	2
No. of glycine residues (shown in triangles)	8
No. of proline residues	6
Total no. of residues	189

**Table 6:** Quality assessment score before and after energy minimization.

Criteria	Before energy minimization	After energy minimization
Energy	- 48361.0 kJ/mol	-11487.9 kJ/mol
Quality factor (ERRAT)	78.453	95.5556
Ramachandran plot (PROCHECK)	90.8%	93.6%
VERIFY 3D	98.41% of the residues have averaged 3D-1D score >= 0.2	96.30% of the residues have averaged 3D-1D score >= 0.2

**Table 7:** T cell epitopes predicted by NetCTL server along with their MHC I binding alleles.

Epitope	Interacting MHC I alleles
QSAQAKNDY	HLA-A∗30 : 02
LTDKNQGFL	HLA-A∗01 : 01
GMEVEITQY	HLA-A∗30 : 02
DSGSNKLPY	HLA-B∗35 : 01
HTDKNNHNP	None
QANQALEQY	HLA-B∗35 : 01, HLA-B∗58 : 01
KQAQGMGKY	HLA-A∗30 : 02, HLA-B∗15 : 01
FAEDNPQEF	HLA-B∗35 : 01, HLA-B∗53 : 01
NQALEQYGY	HLA-A∗30 : 02, HLA-B∗15 : 01
LDDLQFSGY	HLA-A∗01 : 01
AIYHLNVRY	HLA-A∗30 : 02, HLA-A∗32 : 01, HLA-B∗15 : 01, HLA-A∗03 : 01, HLA-A∗11 : 01
DLQRIQGDY	HLA-A∗30 : 02
TVDSGSNKL	None

## Data Availability

The data used to support the findings of this study are included within the article.

## Abbreviations

CASTp: Computed Atlas of Surface Topography of Proteins
CTL: Cytotoxic T lymphocyte
DUF: Domain of unknown functions
GRAVY: Grand average of hydropathicity
HP: Hypothetical protein
IEDB: Immune epitope database
ORF: Open reading frame
pl: Isoelectric point
STD: Sexually transmitted disease
STI: Sexually transmitted infection
UPF: Uncharacterized protein families.
